RETRACTED

# Regulatory B Cell Function Is Suppressed by Smoking and Obesity in *H*. *pylori*-Infected Subjects and Is Correlated with Elevated Risk of Gastric Cancer

**DOI:** 10.1371/journal.pone.0134591

**Published:** 2015-07-30

**Authors:** Guanggang Li, Hasi Wulan, Zongchang Song, Paul A. Paik, Ming L. Tsao, Gary M. Goodman, Paul T. MacEachern, Robert S. Downey, Anna J. Jankowska, Yaron M. Rabinowitz, Thomas B. Learch, David Z. Song, Ji J. Yuan, Shihang Zheng, Zhendong Zheng

**Affiliations:** 1 Affiliated Bayi Brain Hospital, General Hospital of Beijing Military Command, Beijing, 100700, China; 2 Department of Plastic and Reconstructive Surgery, PLA General Hospital, Beijing, 100853, China; 3 Department of Oncology, The 155th Central Hospital of PLA, Kaifeng, 475003, China; 4 Roswell Park Cancer Institute, Buffalo, NY, United States of America; 5 Georgetown University Medical Center, Washington DC, United States of America; 6 University of Maryland Medical Center. Baltimore, MD, United States of America; 7 University Hospital, University of British Columbia, Vancouver, BC, Canada; 8 Department of Gastroenterology, Shengjing Hospital, China Medical University, Shenyang, 110022, China; 9 Department of Medical Oncology, Changzheng Hospital, Second Military Medical University, Shanghai, 200070, China; 10 Department of Oncology, General Hospital of Shenyang Military Area Command, Shenyang, 110840, China; National Cancer Center, JAPAN

## Abstract

*Helicobacter pylori* infection occurs in more than half of the world’s population and is the main cause for gastric cancer. A series of lifestyle and nutritional factors, such as tobacco smoking and obesity, have been found to elevate the risk for cancer development. In this study, we sought to determine the immunological aspects during *H*. *pylori* infection and gastric cancer development. We found that B cells from *H*. *pylori*-infected patients presented altered composition and function compared to uninfected patients. IL-10-expressing CD24^+^CD38^+^ B cells were upregulated in *H*. *pylori*-infected patients, contained potent regulatory activity in inhibiting T cell pro-inflammatory cytokine secretion, and responded directly to *H*. *pylori* antigen stimulation. Interestingly, in *H*. *pylori-*infected smoking subjects and obese subjects, the number of IL-10^+^ B cells and CD24^+^CD38^+^ B cells were reduced compared to *H*. *pylori*-infected asymptomatic subjects. Regulatory functions mediated by CD24^+^CD38^+^ B cells were also impaired. In addition, gastric cancer positive patients had reduced IL-10-producing B cell frequencies after *H*. *pylori*-stimulation. Altogether, these data suggest that in *H*. *pylori*-infection, CD24^+^CD38^+^ B cell is upregulated and plays a role in suppressing pro-inflammatory responses, possibly through IL-10 production, a feature that was not observed in smoking and obese patients.

RETRACTED

## Introduction

*Helicobacter pylori (H*. *pylori)* is a kind of Gram-negative pathogenic bacteria found in more than half of the world’s population and preferentially inhibits the upper gastrointestinal tract, including the stomach epithelium and the duodenum tract[1,2]. Although the vast majority (>80%) of infections are asymptomatic, 10–20% infected subjects will develop peptic ulcers while 1–2% will acquire gastric cancer[3]. The precise mechanism of cancer development as a result of *H*. *pylori* infection is not well defined, but chronic untreated inflammation in the upper gastrointestinal tract is thought to contribute to the continued damage of the stomach epithelium[4,5]. Specifically, inflammation-associated signaling molecules, such as tumor necrosis factor alpha (TNF-a), have been found to promote gastric tumorigenesis and is upregulated in *H*. *pylori* infection[6]. Other pro-inflammatory cytokines secreted by T cells, including IL-2, IL-17, and interferon gamma (IFN-g), are also upregulated in *H*. *pylori* infection and are associated with increased risk of gastric tumorigenesis[7–10]. A series of other factors, such as continuous exposure to tobacco smoking and obesity, are positively correlated with increased gastric cancer risk, though the underlying mechanism is unclear[3,11].

Recently, the role of tolerance-inducing B cells has been characterized in a series of infectious diseases and autoimmune diseases[12]. In mice, CD1d^hi^CD5^+^ B cells have been found to help establish tolerogenic environment in tissues and have a role in preventing autoimmune induction[13]. In humans, CD19^+^CD24^hi^CD38^hi^ B cells have similar tolerance-inducing role in healthy as well as HBV-infected individuals[14]; the onset of autoimmune disease is correlated with loss of regulatory function in this B cell subset[15]. IL-10 is a pleiotropic immunoregulatory cytokine that is capable of inhibiting a series of pro-inflammatory cytokines, including IL-2, IL-17, IFN-g and TNF-a, and is shown to potently suppress the antigen-presenting capacity of antigen presenting cells[16]. Central to all tolerance-inducing B cell subsets, IL-10 production is pivotal to B cell-mediated regulation in suppressing T cell-mediated inflammation[12,17]. The role of B cell-mediated regulation in *H*. *pylori* infection and subsequent induction of gastric cancer, however, was not previously studied.

In this study, we analyzed the B cell composition and cytokine expression profile in *H*. *pylori*-infected subjects. Increased percentages of CD24^+^CD38^+^ B cells and reduced percentages of naïve B cells and resting memory B cells were found in *H*. *pylor*i-infected subjects. The CD24^+^CD38^+^ B cells in *H*. *pylori-infected subjects had* increased percentage of IL-10 production, and had suppressed pro-inflammatory cytokine expression when co-cultured with autologous T cells. *H*. *pylori-s*timulated CD24^+^CD38^+^ B cells from *H*. *pylori-*infected subjects potently secreted IL-10. Interestingly, *H*. *pylori-infected smoking* subjects and obese subects had lowered levels of CD24^+^CD38^+^ B cells. In addition, the CD24^+^CD38^+^ regulatory B cells in smoking and obese subjects were found to exhibit loss of suppressive function when co-cultured with autologous T cells and stimulated reduced levels of IL-10 after direct *H*. *pylori* stimulation. In addition, in smoking and obese patients who later developed gastric cancer, the frequencies of IL-10-secreting B cells were further reduced, compared to the subjects who did not develop gastric cancer. Altogether, these data demonstrated that CD24^+^CD38^+^ B cells were upregulated in *H*. *pylori*-infected and had functionally suppressed T cell inflammatory cytokine production. The CD24^+^CD38^+^ B cells in smoking subjects and obese subjects, however, were refractory to *H*. *pylori*-stimulation, produced less IL-10, and lacked suppressive capacity.

RETRACTED

## Materials and Methods

### Study subjects

Primary peripheral blood samples were obtained from 55 *H*. *pylori*-infected ulcer-free patients, of which 15 are primary consumers of tobacco smoke and 15 are class I obese (30kg/m^2^ < BMI < 35 kg/m^2^) subjects, as well as 15 healthy *H*. *pylori*-uninfected ulcer-free individuals. Individuals with chronic exposure to secondhand smoking were excluded from the study. No significant differences regarding age, sex, and previous infection history between study groups were found. All subjects were followed for 5 years for the cancer development status. All subjects were unrelated individuals from Henan province and its surrounding region. Patients were recruited between Jan 2008 and Dec 2013 from The 155th Central Hospital of PLA in China. Controls were cancer-free individuals randomly selected from a community cancer-screening program for early detection of cancer carried out in the same regions during the same period the patients were recruited. The response rate for both controls and cases was 95%. The selection criteria for healthy controls included cancer-free individuals and frequency matching to cases by sex and age (±5 years). At recruitment, written informed consent was obtained from each subject and personal data such as sex, age, weight, height and tobacco smoking were collected through a questionnaire. Not all subjects’ samples were used in all experiments due to incomplete patient compliance and insufficient cells in some patients. This study was approved by Institutional Review Board of The 155th Central Hospital of PLA.

RETRACTED

### Sample preparation

Peripheral blood mononuclear cells (PBMCs) were isolated from peripheral blood samples with standard Ficoll-Hypaque procedure and frozen immediately at -150°C until use, or used in experiments immediately if noted. Regular culture medium is RPMI-1640 supplemented with 10% fetal bovine serum, 5mL of 100U penicillin/0.1 mg/mL streptomycin, and 5mL of 2mM L-glutamine. Cells were cultured in 5% CO_2_ at 37°C for the stated period of time.

### Cell isolation

T and B cells were isolated using Human T Cell or B cell Negative Selection Kit (Stemcell, Vancouver, Canada), following protocols provided by the manufacturer. The purities of T and B cell isolations were greater than 94% by flow cytometry. For depletion of CD24^+^CD38^+^ B cells in some experiments, purified B cells were stained with PE anti-human CD24 and APC anti-human CD38 for 30 min. The cells were then sent to live cell sorting and CD24^+^CD38^+^ cells were depleted. In the whole B cell setting, total B cells were sent to live cell sorting without the antibodies.

### Flow cytometry

The following anti-human monoclonal antibodies were used: IL-10, TNF-a (eBioscience, San Diego, CA, USA); CD3, CD4, CD19, CD20, CD21, CD24, CD27, CD38 (Biolegend, San Diego, CA, USA); IFN-g (BD Biosciences, San Jose, CA, USA); CD8 (Invitrogen, Grand Island, NY, USA). Purified human IgG (Biolegend, San Diego, CA, USA) was used to block Fc receptors when staining populations containing B cells. For some experiments, phorbol-12-myristate-13-acetate (PMA, Sigma), ionomycin (Sigma, Munich, Germany), or heat-killed *H*. *pylori* (Sigma, Munich, Germany) were used to stimulate cells. GolgiStop and GolgiPlug were added 6h prior to cell harvest for intracellular staining of IL-2, IL-17, IFN-g, TNF-a, and IL-10. FlowJo was used to flow cytometry analysis.

### Luminex assay

IL-2, IL-17, IFN-g, TNF-a and IL-10 from T cells and B cells were quantitatively measured by multiplex Luminex assay following protocols provided by manufacturer with modifications (EMD Millipore, Etobicoke, Canada). A total of 2x10^5^ T cells and/or B cells were plated in each well of 96-well plate (Corning, Tewksbury, MA, USA). For B cell stimulation, heat-killed *H*. *pylori* were added to the B cells, which were plated at the bottom of a 96-well transwell plate (Corning, Tewksbury, MA). For T cell stimulation, the bottom part of the transwell plate was pre-incubated with anti-human CD3 (clone OKT3) overnight and washed, after which purified T cells were transferred into the plate. Human cytokine capture antibody beads were added to the upper chamber of the 96-well transwell plate. Twelve hours later, the beads were harvested, washed and read according to manufacturer’s protocol.

RETRACTED

### Statistical analysis

D’Agostino and Pearson omnibus normality test was used to examine whether the data were normally distributed. One-way analysis of variance (ANOVA) was used for comparisons between multiple groups followed by Dunn’s test. Student’s t test was used for comparisons between two groups. If datasets significantly deviated from normal distribution, nonparametric tests were used. All statistical analyses were done using Prism (GraphPad Software). P<0.05 was considered significant. Results were shown as mean±S.E.M.

## Results

### *H*. *pylori*-infected subjects had altered circulating B cell composition

To analyze the potential changes in the role of B cell responses in *H*. *pylori* infection and how it might be affected by smoking and obesity, 15 healthy *H*. *pylori*-uninfected (*H*. *pylori*-uninfected) volunteers, 20 *H*. *pylori*-infected asymptomatic non-smoking non-obese (asymptomatic) subjects, 15 *H*. *pylori*-infected smoking non-obese (smoking) subjects, and 15 *H*. *pylori*-infected non-smoking obese (obese) subjects were recruited for this study. The demographic and clinical data were summarized in Table 1.

**Table 1:** Demographic and clinical characteristics of study subjects.

	Healthy		H. pylori-infected		P
		Asymptomatic	Smoking	Obese	
N	15	20	15	15	
Female/Male	10/5	13/7	12/3	10/5	N.S.
Age (y)	45.6 (35–55)	44.5 (32–53)	46.2 (33–57)	47.2 (34–56)	N.S.
BMI	21 (18.2–24)	20.3 (18–22.5)	21.4 (18.4–24.6)	31.8 (30.2–34)	< 0.001
Tobacco use					<0.001
None	13	17	0	9	
Past smoker	2	3	0	6	
Current smoker	0	0	15	0	
IMC positive	0	5	7	4	<0.05

Continuous data were represented as mean (range).

Past smoker: smoked before but no longer smoking for at least 1 y.

Current smoker: currently smoking with at least 10 y history.

N.S.: not significant.

Circulating B cells in the peripheral blood of healthy subjects are composed of mainly IgD^+^CD27^-^ naïve B cells and CD21^+^CD27^+^ resting memory B cells, while in chronic infections, there is frequently a decrease in naïve B cells and resting memory B cells, and an increase in CD21^lo^ activated B cells and CD24^+^CD38^+^ B cells[15,18]. We first examined the composition of circulating B cells in *H*. *pylori*-infected subjects. Peripheral blood mononuclear cells (PBMCs) were stained for surface marker expression directly *ex vivo* (Fig 1A). We found that comparing to *H*. *pylori*-uninfected healthy subjects, all *H*. *pylori*-infected groups contained lower percentages of IgD^+^CD27^-^ naïve B cells (P<0.001 for all, Fig 1B and 1C). The percentages of CD21^+^CD27^+^ resting memory B cells were reduced in *H*. *pylori*-infected smoking subjects and obese subjects compared to healthy subjects (P<0.001 for both), and the percentage of CD21^+^CD27^+^ B cells in obese subjects was reduced compared to *H*. *pylori*-infected asymptomatic subjects (P<0.01). Interestingly, the percentages of CD24^+^CD38^+^ B cells were varied among different groups of *H*. *pylori*-infected subjects. *H*. *pylori*-infected asymptomatic subjects contained much higher percentages of CD24^+^CD38^+^ B cells than healthy controls (P<0.001). The percentage of CD24^+^CD38^+^ B cells was reduced in smoking subjects compared to that in asymptomatic subjects (P<0.05), but still higher than that in healthy subjects (P<0.001). In obese subjects, the percentage of CD24^+^CD38^+^ B cells was not significantly different from that in healthy subjects but was reduced from that in asymptomatic subjects (P<0.001).

RETRACTED

**Fig 1:** B cell composition and surface marker expression of H. pylori-infected subjects compared to healthy controls. (A) Gating strategy for B cells in PBMC. All subsequent populations shown were gated accordingly on CD3^-^CD19^+^ live singlet lymphocytes. (B) Representative dot plots depicting IgD vs. CD27, CD27 vs. CD21, and CD38 vs. CD24 expression on B cells in healthy *H*. *pylori*-uninfected subjects (*H*. *pylori*-uninfected, N = 20), *H*. *pylori*-infected non-smoking non-obese asymptomatic (Asymptomatic, N = 15), *H*. *pylori*-infected smoking non-obsese (Smoking, N = 15), and *H*. *pylori*-infected obese non-smoking (Obese, N = 15) subjects. (C) Percentages of IgD^+^CD27^-^ naïve B cells, CD21^+^CD27^+^ classical memory B cells, and CD24^+^CD38^+^ regulatory B cells in study groups. *: P<0.05. **: P<0.01. ***: P<0.001. (Kruskal-Wallis one-way ANOVA and Dunn’s test). For flow cytometry analysis, greater than 10^6^ events in the lymphocyte gate were collected.

### *H*. *pylori*-infected subjects had altered B cell cytokine expression profile

Previously, B cells were found to amplify or suppress immune responses through the production of a series of cytokines with different functions, including pro-inflammatory cytokines such as IL-2, IL-4, IL-6, IL-12, IFN-g and TNF-a, as well as IL-10 and transforming growth factor beta (TGF-b) as regulatory cytokines[19]. Here, we examined the cytokine expression of B cells in study subjects. We found that the *ex vivo* expression of IL-2, IFN-g and TNF-a by B cells were increased in *H*. *pylori*-infected smoking subjects and obese subjects than that in healthy subjects (Fig 2A). No significant differences were found in TGF-b expression.

RETRACTED

**Fig 2:** B cell cytokine expression in H. pylori-infected subjects and in healthy controls. (A) Percentages of total B cells expressing IL-2, IFN-g, TNF-a, and TGF-b in *H*. *pylori-*uninfected (N = 7), *H*.*pylori-*infected asymptomatic (N = 8), *H*. *pylori*-infected smoking (N = 6), and *H*. *pylori*-infected obese (N = 6) subjects under unstimulated (without PMA/ionomycin) condition. (B) Representative dot plots of B cell intracellular cytokine staining without or with PMA/ionomycin stimulation, from an uninfected subject. The cytokine expressions of total B cells minus CD24^+^CD38^+^ B cells (non-CD24^+^CD38^+^ B cells) and that of CD24^+^CD38^+^ B cells were shown separately. (C) Percentages of IL-10-expressing, non-CD24^+^CD38^+^ B cells and CD24^+^CD38^+^ B cells in all study groups, under both unstimulated and PMA/ionomycin stimulated conditions. (D) Numbers of IL-10^+^ B cells in study groups, calculated by the percentage of IL-10-expressing cells in CD24^+^CD38^+^ B cells multiplied by the percentage of CD24^+^CD38^+^ in total B cells (as shown in Fig 1C). *: P< 0.05. **: P<0.01. ***: P<0.001. (Kruskal-Wallis one-way ANOVA and Dunn’s test). For dot plots, 5000 events in each gate were shown.

CD24^+^CD38^+^ B cells have regulatory functions in other studies and had interesting expression levels in different *H*. *pylori*-infected groups (Fig 1C). We examined the intracellular cytokine expression by CD24^+^CD38^+^ B cells. As shown in Fig 2B, the cytokine expression of CD24^+^CD38^+^ B cells were different from non-CD24^+^CD38^+^ B cells (total B cells minus CD24^+^CD38^+^ B cells) in that they did not produce high levels of IFN-g and TNF-a when stimulated with PMA/ionomycin, but expressed very high levels of IL-10, both under unstimulated and stimulated conditions. We compared the production of IL-10 from various B cell subsets and found that CD24^+^CD38^+^ B cells in all study groups secreted much higher IL-10 than non-CD24^+^CD38^+^ B cells, both under unstimulated conditions as well as PMA/ionomycin stimulated conditions (Fig 2C). We thus consider the CD24^+^CD38^+^ fraction as the main IL-10-producing B cell subset. Within the *H*. *pylori*-infected group, asymptomatic subjects had higher percentage of IL-10-expressing cells in CD24^+^CD38^+^ B cells than healthy subjects while *H*. *pylori*-infected obese patients had lower IL-10-expressing cells in CD24^+^CD38^+^ B cells than asymptomatic patients (Fig 2C). We then multiplied the frequency of IL-10^+^ cells in the CD24^+^CD38^+^ B cells with the percentage of CD24^+^CD38^+^ cells in the total B cell to obtain the “number” of IL-10-expressing cells in the B cells, and found that both *H*. *pylori*-infected asymptomatic subjects and smoking subjects had higher levels of IL-10^+^ B cells than healthy subjects (P<0.001 and P<0.01, respectively). Within the *H*. *pylori*-infected group, smoking and obesity significantly lowered the frequencies of IL-10^+^ B cells (P<0.001 for both) from asymptomatic subjects.

RETRACTED

All together, these data demonstrated that regulatory cytokine IL-10 is mainly produced by CD24^+^CD38^+^ B cells and is increased in *H*. *pylori*-infected asymptomatic subjects. Smoking and obesity reduced IL-10 expression in CD24^+^CD38^+^ B cells.

### *H*. *pylori*-infected asymptomatic subjects had more tolerogenic activity mediated by CD24^+^CD38^+^ B cells than smoking and obese subjects

Regulatory B cells were known to inhibit T cell responses in chronic infections, such as hepatitis B infection and human immunodeficiency virus infection[14,20], by establishing tolerogenic environment through IL-10 prior to the induction of inflammation[15,21]. We examined whether the IL-10-producing CD24^+^CD38^+^ B cells had similar regulatory effects in *H*. *pylori*-infection. CD4^+^ T cells co-cultured with autologous CD24^+^CD38^+^-depleted B cells had significantly elevated production of IL-2, IL-17, IFN-g and TNF-a, than CD4^+^ T cells cocultured with whole B cells, in *H*. *pylori*-infected asymptomatic patients (Fig 3A). In smoking subjects and obese subjects, such effect was not observed. Similarly, CD8^+^ T cells from *H*. *pylori*-infected asymptomatic subjects co-cultured with autologous CD24^+^CD38^+^-depleted B cells significantly enhanced IFN-g and TNF-a secretion than those co-cultured with whole B cells (Fig 3B). Again, such effect was not observed in smoking subjects and obese subjects. The suppression of T cell cytokine expression seems to be mediated by CD24^+^CD38^+^ B cells, since lowest cytokine production was observed in CD4^+^ and CD8^+^ T cells co-cultured with CD24^+^CD38^+^ B cells alone. Altogether, these data demonstrated that the CD24^+^CD38^+^ B cells in *H*. *pylori*-infected subjects suppressed CD4^+^ and CD8^+^ T cell pro-inflammatory cytokine production in *H*. *pylori*-infected asymptomatic subjects. Smoking and obesity inhibited regulatory actions of CD24^+^CD38^+^ B cells.

**Fig 3:** T cell cytokine secretion after co-culturing with autologous whole B cells, CD24^+^CD38^+^-depleted B cells, or CD24^+^CD38^+^ B cells. Pure B cells and T cells were isolated from whole PBMCs through magnetic negative selection. Purified B cells were stained with anti-human CD24 and anti-human CD38 antibodies and sent for live cell sorting. The whole B cells, CD24^+^CD38^+^-depleted B cells, or purified CD24^+^CD38^+^ B cells were then co-cultured with autologous T cells in vitro at 1-to-1 ratio for 72h, after which T cells were further separated through magnetic selection into CD4^+^ and CD8^+^ fractions and cultured in the presence of plate-bound anti-CD3 antibody and cytokine capture beads for 6 days. N = 8 for each group. The cytokine productions from (A) CD4^+^ T cells and (B) CD8^+^ T cells were then measured by sensitive luminex assay. *: P< 0.05. **: P<0.01. ***: P<0.001. (Kruskal-Wallis one-way ANOVA and Dunn’s test).

RETRACTED

### IL-10 secretion by CD24+CD38+ B cells upon *H*. *pylori* stimulation in different subjects

We next sought to examine the mechanism of IL-10 upregulation in the B cells of *H*. *pylori*-infected subjects. IL-10 production is pivotal to regulatory B cell function[12,13]. Toll-like receptor signaling is a major IL-10 upregulation mechanism in B cells, and was shown to modulate cytokine expression in *H*. *pylori* infection[22,23]. We tested whether the presence of *H*. *pylori* can directly upregulate IL-10 secretion in CD24^+^CD38^+^ B cells. Purified B cells from PBMCs were cultured in the absence or presence of heat-killed *H*. *pylori* bacterium. After 72h incubation, the secretion of IL-10 in the supernatant was measured by luminex. The B cells were also harvested for intracellular IL-10 staining. As shown in Fig 4A, IL-10 secretion in the supernatant is increased in both *H*. *pylori*-uninfected healthy subjects and *H*. *pylori*-infected non-smoking non-obese asymptomatic subjects after *H*. *pylori*-stimulation (P<0.01 and P<0.05, respectively). Fig 4B shows that the percentage of IL-10-secreting B cells was upregulated in CD24^+^CD38^+^ B cells after *H*. *pylori* stimulation in healthy and asymptomatic subjects (P<0.001 and P<0.05, respectively). In contrast, the concentration of IL-10 in the supernatant and the percentage of IL-10-producing CD24^+^CD38^+^ B cells from *H*. *pylori*-infected smoking subjects and obese subjects were not significantly increased after *H*. *pylori*-infection. These data demonstrated that smoking and obesity had impaired the induction of IL-10 from B cells after *H*. *pylori* stimulation, and suggested that in part, the loss of regulatory function of CD24^+^CD38^+^ B cells from smoking subjects and obese subjects was possibly due to an inability to upregulate IL-10 secretion in response to bacterial antigen stimulation (See discussion).

**Fig 4:** CD24^+^CD38^+^ B cell responses to bacterial antigen stimulation in different study groups. Total B cells were isolated from PBMCs by negative selection and then cultured in the absence or presence of heat-killed *H*. *pylori* bacterium, together with IL-10 capture beads. After 72h incubation, the secretion of IL-10 in the supernatant was collected by capture beads and measured by luminex assay. The B cells were also harvested for intracellular IL-10 staining. N = 8 for every group. (A) Secreted IL-10 concentration in the supernatant. (B) Percentage of IL-10^+^ cells in CD24^+^CD38^+^ B cells at the end of the 72h incubation. *: P< 0.05. **: P<0.01. ***: P<0.001. (Student’s *t* test).

RETRACTED

### Gastric cancer-positive patients in the *H*. *pylori*-infected smoking and *H*. *pylori*-infected obese groups had lower frequencies of IL-10^+^ B cells

Smoking and obesity were known to increase the risk for gastric cancer development in *H*. *pylori*-infected subjects. Since smoking and obesity also suppressed normal regulatory B cell functions, we examined whether these two phenomena were linked. We found that in smoking subjects and obese subjects, those who became positive for gastric cancer status had significantly lower frequencies of IL-10^+^ cells in CD24^+^CD38^+^ B cells after *H*. *pylori* stimulation than those who remained negative for gastric cancer development (Fig 5A. P<0.05 for both). On the other hand, we did not find that cancer positive and cancer negative patients were significantly different in terms of their frequencies of CD24^+^CD38^+^ B cells in total B cells (Fig 5B). No *H*. *pylori-*infected asymptomatic patients in this study became gastric cancer positive.

**Fig 5:** Frequencies of IL-10^+^ B cells and CD24^+^CD38^+^ B cells in study subjects with or without gastric cancer development. Patients’ gastric cancer status was tracked for 5 years after initial sample collection. (A) The frequencies of IL-10^+^ cells in CD24^+^CD38^+^ B cells after direct *H*. *pylori* stimulation in *H*. *pylori*-infected smoking subjects and obese subjects (B) The percentages of CD24^+^CD38^+^ B cells in total B cells in *H*. *pylori*-infected smoking subjects and obese subjects. N = 8 for every group. *: P< 0.05. (Student’s *t* test).

## Discussion

*H*. *pylori* infection is the major cause of the development of gastric cancer. Although the majority of infections were asymptomatic and treatable, a subset of subjects fails treatment and progress to gastric cancer. In addition, smoking and obesity increase the risk of cancer development while the mechanisms are not entirely clear. In this study, we first observed an alteration in circulating B cell composition in *H*. *pylori*-infected asymptomatic subjects compared to uninfected healthy subjects, with a reduction of IgD^+^CD27^-^ naive B cells and an upregulation of CD24^+^CD38^+^ B cells. The CD24^+^CD38^+^ B cells were also found to be the main IL-10-secreting B cell subset. We then performed T cell-B cell coculture experiments and found that T cells in CD24^+^CD38^+^ B cell-depleted co-cultures secreted higher levels of proinflammatory cytokines than T cells co-cultured with whole B cells, while T cells cocultured with CD24^+^CD38^+^ B cells only had the lowest pro-inflammatory cytokine production. Furthermore, we discovered that the presence of *H*. *pylori* could directly enhance IL-10-expression from CD24^+^CD38^+^ B cells. Together, these data demonstrated that *H*. *pylori*-infected subjects had upregulated frequencies of circulating CD24^+^CD38^+^ B cells, which expressed high levels of IL-10 and exhibited regulatory function. Interestingly, in *H*. *pylori*-infected smoking subjects and obese subjects, the circulating CD24^+^CD38^+^ B cells were reduced in frequency compared to *H*. *pylori*-infected asymptomatic subjects, were unable to suppress T cell pro-inflammatory cytokine production in co-culture experiments, and did not significantly upregulate IL-10 expression after *H*. *pylori* stimulation. In addition, we followed the subjects for five years and subsequently found that compared to gastric cancer-positive patients, gastric cancer-negative patients had more IL-10 production after *H*. *pylori* stimulation. Chronic cell destruction and tissue lesions in persistent *H*. *pylori* infection were major contributing factors to gastric cancer development[24]. From results presented in this paper, it is possible that increased IL-10-expression by B cells may protect the *H*. *pylori*-infected subjects by reducing T cell-mediated inflammation and limiting tissue lesions, but in smoking subjects and obese subjects, the B cell-mediated tissue protection was not present. More studies are needed in the future to examine whether the presence of IL-10^+^ B cells is correlated with reduced tissue lesions in *H*. *pylori* infection. This, however, was not feasible in this study since it requires gastric tissue samples.

RETRACTED

It has been reported that tobacco smoking is associated with increased oxidative stress and pro-inflammatory cytokine release, possibly due to smoking-induced tissue damage[25,26]. Obesity is also associated with increased low-grade, chronic inflammation[27]. In this study, we found that *H*. *pylori*-infected smoking subjects and obese subjects had less IL-10^+^ B cells than *H*. *pylori*-infected asymptomatic subjects. Subsequently, unlike that in asymptomatic subjects, presence of CD24^+^CD38^+^ B cells from smoking subjects and obese subjects in the T cell-B cell co-culture did not reduce T cell pro-inflammatory cytokine production. The reduction in IL-10 production and the lack of regulatory function in B cells may have resulted from the overall increased inflammatory state in smoking and obesity. Indeed, our data showed that B cells from *H*. *pylori*-infected smoking and obese subjects, but not those from asymptomatic subjects, had higher IL-2, IFN-g, and TNF-a production than B cells from uninfected healthy subjects, suggesting a skewing toward a more proinflammatory phenotype. At the same time, exposure to chronic smoking and obesity are known to associate with increased gastric cancer risk. Together, these data suggest that a more pro-inflammatory immune profile in smoking and obese population may contribute to gastric cancer development.

Due to the lack of regulatory B cell-specific transcription factors and surface molecules, various non-specific sets of surface markers, including CD1d^hi^CD5^+^, CD19^+^CD24^hi^CD38^hi^, and CD19^+^TIM-1^+^, had been used in previous studies to denote B cells with regulatory activities [15,22,28,29]. In this study, we focused on CD24^+^CD38^+^-expressing B cells because we found that IL-10, a pivotal cytokine in regulatory B cell function, is enriched in this subset, and Fig 3 has demonstrated that this subset had regulatory activity in suppression T cell cytokine production. This choice of surface markers, however, did have caveats, since CD19^+^CD24^hi^CD38^hi^ were previously described as immature/transitional B cells[30,31]. B cells can act as important antigen-presenting cells and were found to support T cell subpopulation differentiation and maintenance[32]. At this point, it is unknown whether CD24^+^CD38^+^ B cells in our study were potentially immature/transitional B cells, which may be less effective at antigen presentation. To prevent this problem, we compared whole B cells with CD24^+^CD38^+^-depleted B cells (both groups with mature B cells capable of “normal” antigen presentation), and subsequently re-stimulated T cells with anti-CD3 for direct T cell receptor (TCR) activation. Although we also included a CD24^+^CD38^+^ B cell-only group in the co-culture experiment, and found that T cells in these co-cultures had significantly reduced proinflammatory cytokine production than T cells in CD24^+^CD38^+^ B cell-depleted cocultures, we cannot exclude the possibility that this reduction were due to potentially defective antigen presentation during the co-culture, prior to direct TCR activation.

The role of regulatory cells in the immune system was frequently seen as a double-edged sword in chronic infections. On one hand, the suppression of inflammation by regulatory T cells and B cells can prevent excessive tissue damage mediated by the immune system. On the other hand, regulatory T cell and B cell-mediated inhibition of immune activation were thought to contribute to pathogen persistence, effector T cell exhaustion, and lowered ability to clear infections. Previously, IL-10-secretion in B cells was found to contribute to *Salmonella typhimurium* and mouse mammary tumor virus persistence in mice and HIV persistence in humans[20,33,34]. In this study, we found that addition of *H*. *pylori* could directly activate B cell IL-10 production, but it is unclear how the upregulation of CD24^+^CD38^+^ B cells and IL-10 secretion can affect *H*. *pylori* infection. Whether regulatory B cells contribute to bacterial persistence in *H*. *pylori* infection requires more studies.

RETRACTED

## References

[1] MalfertheinerP, SelgradM. Helicobacter pylori. Curr Opin Gastroenterol. 2014;30: 589–595. Available: http://www.hubmed.org/display.cgi?uids=25268839 10.1097/MOG.0000000000000128 25268839

[2] AlbuquerqueA, RiosE, CarneiroF, MacedoG. Evaluation of clinico-pathological features and Helicobacter pylori infection in gastric inflammatory fibroid polyps. Virchows Arch. 2014;465: 643–647. Available: http://www.hubmed.org/display.cgi?uids=25257403 10.1007/s00428-014-1659-6 25257403

[3] CarcasLP. Gastric cancer review. J Carcinog. 2014;13: 14 Available: http://www.hubmed.org/display.cgi?uids=25589897 10.4103/1477-3163.146506 25589897PMC4278094

[4] RheeK-H, ParkJ-S, ChoM-J. Helicobacter pylori: bacterial strategy for incipient stage and persistent colonization in human gastric niches. Yonsei Med J. 2014;55: 1453–1466. Available: http://www.hubmed.org/display.cgi?uids=25323880 10.3349/ymj.2014.55.6.1453 25323880PMC4205683

[5] QadriQ, RasoolR, GulzarGM, NaqashS, ShahZA. H. pylori infection, inflammation and gastric cancer. J Gastrointest Cancer. 2014;45: 126–132. Available: http://www.hubmed.org/display.cgi?uids=24557546 10.1007/s12029-014-9583-1 24557546

[6] OshimaH, IshikawaT, YoshidaGJ, NaoiK, MaedaY, NakaK, et al TNF-α/TNFR1 signaling promotes gastric tumorigenesis through induction of Noxo1 and Gna14 in tumor cells. Oncogene. 2014;33: 3820–3829. Available: http://www.hubmed.org/display.cgi?uids=23975421 10.1038/onc.2013.356 23975421

[7] GrayBM, FontaineCA, PoeSA, EatonKA. Complex T cell interactions contribute to Helicobacter pylori gastritis in mice. Infect Immun. 2013;81: 740–752. Available: http://www.hubmed.org/display.cgi?uids=23264048 10.1128/IAI.01269-12 23264048PMC3584856

[8] ShiomiS, ToriieA, ImamuraS, KonishiH, MitsufujiS, IwakuraY, et al IL-17 is involved in Helicobacter pylori-induced gastric inflammatory responses in a mouse model. Helicobacter. 2008;13: 518–524. Available: http://www.hubmed.org/display.cgi?uids=19166417 10.1111/j.1523-5378.2008.00629.x 19166417PMC2631559

RETRACTED

[9] KopitarAN, StegelV, TepesB, GubinaM, NovakovićS, IhanA. Specific T cell responses to Helicobacter pylori predict successful eradication therapy. J Infect. 2007;54: 257–261. Available: http://www.hubmed.org/display.cgi?uids=16824607 1682460710.1016/j.jinf.2006.05.009

[10] EppleinM, XiangY-B, CaiQ, PeekRM, LiH, CorreaP, et al Circulating cytokines and gastric cancer risk. Cancer Causes Control. 2013;24: 2245–2250. Available: http://www.hubmed.org/display.cgi?uids=24052422 10.1007/s10552-013-0284-z 24052422PMC3828746

[11] PourhoseingholiMA, VahediM, BaghestaniAR. Burden of gastrointestinal cancer in Asia; an overview. Gastroenterol Hepatol Bed Bench. 2015;8: 19–27. Available: http://www.hubmed.org/display.cgi?uids=25584172 25584172PMC4285928

[12] MauriC, BosmaA. Immune regulatory function of B cells. Annu Rev Immunol. 2012;30: 221–241. 10.1146/annurev-immunol-020711-074934 22224776

[13] CandandoKM, LykkenJM, TedderTF. B10 cell regulation of health and disease. Immunol Rev. 2014;259: 259–272. Available: http://www.hubmed.org/display.cgi?uids=24712471 10.1111/imr.12176 24712471PMC4049540

[14] DasA, EllisG, PallantC, LopesARR, KhannaP, PeppaD, et al IL-10-producing regulatory B cells in the pathogenesis of chronic hepatitis B virus infection. J Immunol. 2012;189: 3925–3935. 10.4049/jimmunol.1103139 22972930PMC3480715

[15] BlairPA, NoreñaLY, Flores-BorjaF, RawlingsDJ, IsenbergDA, EhrensteinMR, et al CD19(+)CD24(hi)CD38(hi) B cells exhibit regulatory capacity in healthy individuals but are functionally impaired in systemic Lupus Erythematosus patients. Immunity. 2010;32: 129–140. 10.1016/j.immuni.2009.11.009 20079667

[16] OuyangW, RutzS, CrellinNK, ValdezPA, HymowitzSG. Regulation and functions of the IL-10 family of cytokines in inflammation and disease. Annu Rev Immunol. 2011;29: 71–7109. 10.1146/annurev-immunol-031210-101312 21166540

[17] RosserEC, BlairPA, MauriC. Cellular targets of regulatory B cell-mediated suppression. Mol Immunol. 2014;62: 296–304. Available: http://www.hubmed.org/display.cgi?uids=24556109 10.1016/j.molimm.2014.01.014 24556109

[18] MoirS, BucknerCM, HoJ, WangW, ChenJ, WaldnerAJ, et al B cells in early and chronic HIV infection: evidence for preservation of immune function associated with early initiation of antiretroviral therapy. Blood. 2010;116: 5571–5579. Available: http://www.hubmed.org/display.cgi?uids=20837780 10.1182/blood-2010-05-285528 20837780PMC3031405

RETRACTED

[19] LundFE. Cytokine-producing B lymphocytes-key regulators of immunity. Curr Opin Immunol. 2008;20: 332–338. Available: http://www.hubmed.org/display.cgi?uids=18417336 10.1016/j.coi.2008.03.003 18417336PMC2474694

[20] LiuJ, ZhanW, KimCJ, ClaytonK, ZhaoH, LeeE, et al IL-10-producing B cells are induced early in HIV-1 infection and suppress HIV-1-specific T cell responses. PLoS One. 2014;9 10.1371/journal.pone.0089236 PMC393171424586620

[21] MatsushitaT, YanabaK, BouazizJD, FujimotoM, TedderTF. Regulatory B cells inhibit EAE initiation in mice while other B cells promote disease progression. J Clin Invest. 2008;118: 3420–3430. 10.1172/JCI36030 18802481PMC2542851

[22] YanabaK, BouazizJ-D, MatsushitaT, TsubataT, TedderTF. The development and function of regulatory B cells expressing IL-10 (B10 cells) requires antigen receptor diversity and TLR signals. J Immunol. 2009;182: 7459–7472. 10.4049/jimmunol.0900270 19494269PMC3733128

[23] KäbischR, Mejías-LuqueR, GerhardM, PrinzC. Involvement of Toll-like receptors on Helicobacter pylori-induced immunity. PLoS One. 2014;9 Available: http://www.hubmed.org/display.cgi?uids=25153703 10.1371/journal.pone.0104804PMC414322225153703

[24] YamaokaY, GrahamDY. Helicobacter pylori virulence and cancer pathogenesis. Futur Oncol. 2014;10: 1487–1500. Available: http://www.hubmed.org/display.cgi?uids=25052757 10.2217/fon.14.29PMC419705925052757

[25] Van der VaartH, PostmaDS, TimensW, ten HackenNHT. Acute effects of cigarette smoke on inflammation and oxidative stress: a review. Thorax. 2004;59: 713–21. 10.1136/thx.2003.012468 15282395PMC1747102

[26] ArnsonY, ShoenfeldY, AmitalH. Effects of tobacco smoke on immunity, inflammation and autoimmunity. J Autoimmun. 2010;34 10.1016/j.jaut.2009.12.003 20042314

[27] GregorMF, HotamisligilGS. Inflammatory mechanisms in obesity. Annu Rev Immunol. 2011;29: 415–45. 10.1146/annurev-immunol-031210-101322 21219177

[28] XiaoS, BrooksCR, ZhuC, WuC, SweereJM, PeteckaS, et al Defect in regulatory B-cell function and development of systemic autoimmunity in T-cell Ig mucin 1 (Tim-1) mucin domain-mutant mice. Proceedings of the National Academy of Sciences. 2012 pp. 12105–12110. 10.1073/pnas.1120914109 PMC340973922773818

[29] DingQ, YeungM, CamirandG, ZengQ, AkibaH, YagitaH, et al Regulatory B cells are identified by expression of TIM-1 and can be induced through TIM-1 ligation to promote tolerance in mice. J Clin Invest. 2011;121: 3645–3656. 10.1172/JCI46274 21821911PMC3163958

[30] SimsGP, EttingerR, ShirotaY, YarboroCH, IlleiGG, LipskyPE. Identification and characterization of circulating human transitional B cells. Blood. 2005;105: 4390–4398. 10.1182/blood-2004-11-4284 15701725PMC1895038

RETRACTED

[31] PalanichamyA, BarnardJ, ZhengB, OwenT, QuachT, WeiC, et al Novel human transitional B cell populations revealed by B cell depletion therapy. J Immunol. 2009;182: 5982–5993. 10.4049/jimmunol.0801859 19414749PMC2746373

[32] BatistaFD, HarwoodNE. The who, how and where of antigen presentation to B cells. Nat Rev Immunol. 2009;9: 15–27. 10.1038/nri2454 19079135

[33] NevesP, LampropoulouV, Calderon-GomezE, RochT, StervboU, ShenP, et al Signaling via the MyD88 adaptor protein in B cells suppresses protective immunity during Salmonella typhimurium infection. Immunity. 2010;33: 777–790. Available: http://www.hubmed.org/display.cgi?uids=21093317 10.1016/j.immuni.2010.10.016 21093317

[34] KaneM, CaseLK, KopaskieK, KozlovaA, MacDearmidC, ChervonskyA V, et al Successful transmission of a retrovirus depends on the commensal microbiota. Science (80-). 2011;334: 245–249. Available: http://www.hubmed.org/display.cgi?uids=21998394 10.1126/science.1210718 21998394PMC3519937

